# Human fetal skin-derived stem cell secretome enhances radiation-induced skin injury therapeutic effects by promoting angiogenesis

This article has been retracted.

**DOI:** 10.1186/s13287-019-1456-x

**Published:** 2019-12-16

**Authors:** Xiaoli Rong, Jiannan Li, Yanyan Yang, Liyan Shi, Tiechao Jiang

**Affiliations:** 1 The Scientific Research Center, China-Japan Union Hospital of Jilin University, 126 Xiantai St., Changchun, 130033 Jilin China; 2 Department of General Surgery, The Second Hospital of Jilin University, 218 Ziqiang St., Changchun, 130041 Jilin China; 3 Department of Ultrasound, China-Japan Union Hospital of Jilin University, 126 Xiantai St., Changchun, 130033 Jilin China; 4 Department of Cardiology, China-Japan Union Hospital of Jilin University, 126 Xiantai St., Changchun, 130033 Jilin China; 5 Jilin Provincial Cardiovascular Research Institute, 126 Xiantai St., Changchun, 130033 Jilin China

**Keywords:** hFSSC, Secretome, Radiation skin injury, Angiogenesis

## Abstract

**Background:**

Radiation dermatitis is a refractory skin injury caused by radiotherapy. Human fetal skin-derived stem cell (hFSSC) is a preferable source for cell therapy and skin tissue regeneration. In the present study, we investigated the repair effect of using hFSSC secretome on a radiation skin injury model in rats.

**Methods:**

We prepared the hFSSC secretome and studied its effects on the proliferation and tube formation of human umbilical vein endothelial cell (HUVEC) in vitro. Furthermore, we used a Sr-90 radiation-induced skin injury model of rats and evaluated the effects of hFSSC secretome on radiation skin injury in vivo.

**Results:**

The results showed that hFSSC secretome significantly promoted the proliferation and tube formation of HUVEC in vitro; in addition, hFSSC secretome-treated rats exhibited higher healing quality and faster healing rate than the other two control groups; the expression level of collagen type III α 1 (Col3A1), transforming growth factor β3 (TGF-β3), angiotensin 1 (Ang-1), angiotensin 2 (Ang-2), vascular endothelial growth factor (VEGF), and placental growth factor (PLGF) was significantly increased, while collagen type I α 2 (Col1A2) and transforming growth factor β1 (TGF-β1) were decreased in hFSSC secretome group.

**Conclusions:**

In conclusion, our results provided the first evidence on the effects of hFSSC secretome towards radiation-induced skin injury. We found that hFSSC secretome significantly enhanced radiation dermatitis angiogenesis, and the therapeutic effects could match with the characteristics of fetal skin. It may act as a kind of novel cell-free therapeutic approach for radiation-induced cutaneous wound healing.

## Background

Radiation is a kind of essential modality for the treatment of malignancy, with over 60% of cancer patients receiving radiotherapy [1]. However, variable degrees of damage often occur in skin tissues during radiotherapy [2]. When intolerable doses of radiation are administered, serious radiation-induced skin injuries can cause severe pain, secondary infection, ulceration, and even necrosis [3]. Therefore, radiation-induced skin injury remains a serious concern, which may limit the duration and dose of radiation treatment [4].

Recent studies have shown stem cells to be a promising strategy to treat refractory skin damage [5]. In the present study, the human fetal skin-derived stem cell (hFSSC), which is the early stage of adult stem cells derived from 8 to 12 weeks fetus of spontaneous abortion, was used [6]. Fetal skin tissue which is donated with consent for research is processed in vitro, confirming cell function without genetic abnormality and contamination [7]. Fetal tissue contains a large number of stem cells and progenitor cells for development, making it helpful for the treatment of skin injuries [8]. Furthermore, fetal tissue cells are easier to culture and can proliferate more readily than comparable adult tissue cells [9]. Fetal tissue cells are also less likely to be rejected by transplant recipients, as these cells are less antigenic, expressing human leukocyte antigen G (HLA-G) for immune tolerance during pregnancy [10]. Because of these special features, the fetal tissue cells can facilitate the engraftment process of skin repair-assisted materials in vivo and may provide beneficial effects against skin injury [11]. Fetal skin in the uterus is observed to lead to scarless tissue repair rapidly, while adult skin wounds heal more slowly with scar formation to restore tissue integrity [12]. The unique properties of fetal cells, including fetal extracellular matrix (ECM), cytokine and growth factor profile (e.g., transforming growth factor β, TGF-β), and homebox gene expression, contribute to wound scarless repair [13, 14].

Recent studies have revealed that implanted stem cells cannot survive for long, and the benefits of mesenchymal stem cell (MSC) therapy could be due to the large amount of biologically active factors they produce, which play an essential role in the regulation of tissue regeneration [15, 16]. MSC secretome derivatives may present considerable advantages over their parental cells, such as easier to be manufactured, less immunogenic, and more convenient to be stored and handled [17]. Therefore, as a kind of cell-free reagent, MSC secretome derivatives possess significant clinical utility. A study has demonstrated that the secretome of MSC isolated from fetal rather than adult skin increased the angiogenesis which is beneficial for wound healing [18]. However, the administration of hFSSC secretome in radiation-induced skin injury has not been reported, and the potential therapeutic mechanism remains unclear.

The present study was designed to investigate whether hFSSC secretome is effective to treat the radiation-induced injury skin in rats. Furthermore, we investigated the effects of hFSSC secretome on angiogenesis both in vitro and in vivo. Our preliminary study clearly demonstrated that compared with human umbilical cord mesenchymal stem cell (hUCMSC), the administration of hFSSC secretome significantly promoted the angiogenesis and fetal-like skin regeneration. Scheme 1 shows the mechanisms of hFFSC secretome in wound healing of our study.

**Scheme 1:** The mechanisms of hFFSC secretome in wound healing

## Materials and methods

### Cell culture and secretome preparation

hFSSC and hUCMSC were provided by Rongyi Stem Cell Medical Technology Co., Ltd. (Changchun, China). Human ethics approval was obtained from the Clinical Research Ethics Committee of the Jilin University (reference no. 201801078). The informed written consent form was approved by the Clinical Research Ethics Committee and signed by the donor before sample collection. P3–5 lines of hFSSCs were used in the experiments. Cell secretome was collected as reported in a previous study [19]. Briefly, cells were cultured and reached 80% confluence, then placed in serum-free medium (SFM; Invitrogen, Shanghai, China), incubated in 5% CO_2_ in a humidified condition. After 24 h, the conditioned medium was collected and centrifuged to purify for 10 min at 4 °C, 4000*g*. After that, 10 ml conditioned medium was re-centrifuged with Amicon Ultra Centrifugal Filters (Millipore Corp, Billerica, MA, USA) at 4 °C, 4000*g*, 2 h. Then, 300–500 μl supernatant solution was collected as cell-free secretome each time. The protein content was measured using the BCSA kit (Thermo Scientific, Rockford, IL, USA) according to the manufacturer’s instruction. HUVEC was acquired from Dr. Chen in our lab, and cultured reference to above methods.

### Immunofluorescence staining

hFSSCs of P3 and HUVECs (cultured by secretome 100 μg/ml) were incubated in 24-well plate for 24 h. When cells reached 70% confluence, they were incubated with 4% paraformaldehyde for 10 min and incubated with 1% bovine serum albumin (BSA; Biosharp, Hefei, China) for 30 min. Then, hFSSCs were incubated with antibodies against CD73, CD90, CD105, Oct4, Sox2 (1:100 dilution, Abcam, Cambridge, UK), and isotype-matched rabbit or mouse IgG/IgM (1:100 dilution, Abcam, Cambridge, UK) which served as the negative controls, and HUVECs were incubated with antibodies against Ki-67 (1:100 dilution, BD Biosciences, Franklin Lakes, NJ, USA) and secondary antibody (anti-rabbit IgG, 1:500 dilution, Abcam, Cambridge, UK). The nuclei were labeled with DAPI (Thermo Scientific, Waltham, USA). Then, the intensity was examined by fluorescence microscopy (EVOS, Thermo Scientific, Waltham, USA), and positive cells were analyzed in ten random optical fields.

### Flow cytometry analysis of surface markers

Flow cytometry (FACSCalibur, Becton Dickinson, CA, USA) was used to detect hFSSCs’ surface antigens (105 cells per marker). Briefly, hFSSCs at approximately 90% confluency were trypsinized and fixed in 3.7% formaldehyde solution. All antibodies were diluted (1:100) with 1% bovine serum albumin (BSA). Cells were labeled with FITC-conjugated anti-CD73, CD90, CD105, Oct4, and Sox2 (BioLegend, San Diego, CA, USA) at 4 °C for 1 h. Appropriate isotype-matched antibodies were used as negative controls (BD Biosciences, San Jose, CA, USA). Data from 10,000 viable cells were acquired. List mode files were analyzed by FCS Express software (BD Biosciences).

### Cell proliferation assay

HUVECs were cultured until cells grew to 80% confluence, then seeded in 96-well plates at a density of 3000 cells per well, supplemented with hUCMSC secretome, hFSSC secretome (100 μg/ml), or SFM (Invitrogen, Shanghai, China), incubated at 37 °C with 5% CO_2_ for 5 days. Cell viability was examined by CCK-8 (Sigma, San Francisco, USA), and corresponding OD value measured on each day at the 490 nm wavelength.

### Tube formation assay

The taken pre-cooled Matrigel (Sigma, San Francisco, USA) 250 μl was added to each well of a 24-well plate at 37 °C for 30 min. Then, 6 × 10^4^ HUVECs were seeded on the surface of the Matrigel and supplemented with hUCMSC secretome, hFSSC secretome (100 μg/ml), or SFM (Invitrogen, Shanghai, China) incubated at 37 °C with 5% CO_2_ for 6 h (Additional file 1). Tube formation was observed with a microscope (× 100) with a digital camera (EVOS, Life Technologies, Foster City, CA, USA). Total branch points and tube lengths/field were calculated by Image J.

### Animals and treatments

The animal model was made according to previously published methods with some modifications [4]. All the protocols and procedures were approved by the Animal Experiment Ethic Committee of Jilin University (approval no. 20180143). Rats (8-week female SD) were anesthetized with an intraperitoneal injection of 10% chloral hydrate (500 μl/100 g). The hair on rat buttock skin was shaved using a razor, and then, a 3-cm-thick piece of lead was used to shield the rats and localize the radiation field (2 cm × 2 cm). The buttock skin of rats was irradiated with a β-ray beam (Sr90), the irradiation dose of 50 Gy (with almost 100% successful rate) in an area of 2 cm × 2 cm in 30 min. The irradiated animals were randomly divided into three groups with ten rats per group: SFM (negative control), hUCMSC secretome (positive control), and hFSSC secretome. Rats were administered secretome through subcutaneous injection (1 mg secretome per 1 ml injection) or SFM (1 ml) once a week. Rats were euthanized at 7 weeks after radiation, and the wound healing tissues were collected for use. The wound area was analyzed by Adobe Photoshop CS6. Wound closure rate (%) = [(wound area on original − wound area on *N*th day)/wound area on original] × 100.

### Skin histological analysis

Cross sections of healed tissue were taken, fixed in 4% formaldehyde, and embedded in paraffin. Skin tissue sections with 4 μm thickness were used for staining. Tissue cross sections were stained with hematoxylin and eosin according to the manufacturer’s protocol. Immunohistochemistry (IHC) was measured with the kit (Maixin KIT-9710, Fuzhou, China) in accordance with the manufacturer’s instructions. The primary antibody was α smooth muscle actin (α-SMA) (ab5694, Abcam, Cambridge, UK), and the second antibody was biotinylated goat-anti-rabbit IgG, photographed by the optical microscope (Olympus, Tokyo Metropolitan, Japan). The number of cutaneous appendages and vessel was determined by manually counting in ten random optical fields.

### Real-time PCR assay

Total RNA from wound healing tissue was extracted with Trizol (Invitrogen, Shanghai, China) according to the manufacturer’s protocol. SYBR Green I dye was used for reverse transcription in an ABI 7500 fluorescence quantitative PCR instrument, and the mRNA levels of collagen type I α 2 (Col1A2), collagen type III α 1 (Col3A1), TGF-β1, TGF-β3, angiotensin 1 (Ang-1), angiotensin 2 (Ang-2), vascular endothelial growth factor (VEGF), and placental growth factor (PLGF) were measured, and the primers are added in Additional file 2: Table S1. Thermocycler conditions are as follows: initial step at 95 °C for 2 min, followed by 40 cycles at 95 °C for 15 s and 60 °C for 1 min. Expression levels were recorded as cycle threshold (Ct). Data were acquired using the 7500 Software (Applied Biosystems Life Technologies, Foster City, CA, USA). All reactions were performed in triplicate, and the data were analyzed using the 2^-ΔΔCt^ method.

### Western blot

Proteins were extracted from the healed skin tissue in the lysis buffer. Protein samples in SDS sample buffer were heated at 95 °C for 10 min and separated on SDS-polyacrylamide gels. Resolved proteins were then electro blotted onto nitrocellulose membranes and probed with antibody against Col1A2, Col3A1, TGF-β1, TGF-β3, Ang-1, Ang-2, VEGF, PLGF, and glyceraldehyde-3-phosphate dehydrogenase (GAPDH) (1:1000 dilution, Abcam, Cambridge, UK) overnight at 4 °C. These were followed by secondary antibodies HRP-conjugated goat anti-rabbit IgG (1:1000 dilution, Abcam, Cambridge, UK) and visualized by chemiluminescent detection according to the manufacturer’s instructions (Immobilon western chemiluminescent HRP substrate, Millipore).

### Statistical analysis

Statistical analysis was performed using Prism 6 (Graph Pad software) and Image J. One-way ANOVA with Dunnett’s multiple comparisons test was used to test for statistically significant differences. All quantitative data were given as the mean ± SD for at least three independent experiments. *p* < 0.05 was considered to be statistically significant.

## Results

### Immunofluorescence staining analysis of hFSSC markers

The antigen profiles of hFSSCs after three passages in culture were analyzed by immunofluorescence staining. The results showed that hFSSCs were strongly positive for surface markers, such as CD73, CD90, CD105, Oct4, and Sox2 (Fig. 1). Characterization work confirms that besides expressing classical MSC markers (such as CD73, CD90, and CD105), the hFSSCs also expressed some key markers of embryonic stem cells (such as Oct4 and Sox2).

**Fig. 1:** The characterization of hFSSCs. **a** Cells at passage 3 were used, and the conjugated fluorescent dyes are as follows: CD73, CD90, CD105, Oct4, and Sox2. **b** Flow cytometry analysis of hFFSCs. Expressions of indicated antigen (CD73, CD90, CD105, Oct4, and Sox2) are shown in red histograms in contrast to isotype controls (gray histograms). Note that bar = 200 μm; hFSSC, human fetal skin stem cell

### hFSSC secretome promoted HUVEC proliferation and tube formation in vitro

As shown in Fig. 2a, b, we found that compared to the other two control groups, hFSSC secretome had the highest percentage of Ki-67-positive cells in HUVEC (SFM 15.2%, hUCMSC secretome 72.3%, and hFSSC secretome 88.4%). CCK-8 results showed that the growth rates of HUVEC in the hFSSC secretome group were significantly increased compared to the other two control groups (Fig. 2c). The steepest slope occurred between 2 and 4 days; thereafter, the OD value came to the platform period along with increasing time. To investigate the role of hFSSC secretome in the regulation of tube formation, HUVEC tube formation was studied by growing cells in Matrigel. We found that hFSSC secretome group promoted tube formation significantly (Fig. 3a). Moreover, the branching point/field of hFSSC secretome group was the most (*p* < 0.001), and tube length was longer in hFSSC secretome group than that in the other two control groups (Fig. 3b, c; *p* < 0.001).

**Fig. 2:** Effects of the hFSSC secretome on proliferation of HUVEC. **a** Immunofluorescent staining of antibody on HUVEC. **b** Percentages of Ki-67-positive cells in HUVEC. **c** The proliferation curves of HUVEC using hFSSC secretome. Note that hFSSC secretome group showed the highest percentage of Ki-67-positive cells and proliferation rate compared to the other two groups. HUVEC, human umbilical vascular endothelial cell; SFM, serum-free medium; hUCMSC, human umbilical cord mesenchymal stem cell; hFSSC, human fetal skin stem cell. *p < 0.05, **p < 0.01, ***p < 0.001, when compared to SFM; bar = 200 μm; data, *n* = 3; mean ± SD

**Fig. 3:** Effects of hFSSC secretome on tube formation by HUVEC. **a** HUVEC tube formation was studied by growing cells in Matrigel in SFM containing 100 μg/ml hUCMSC or hFSSC secretome for 6 h. Bar = 1 mm. **b** Total branch points/field and **c** tube lengths/field of HUVEC following growth in SFM containing 100 μg/ml hUCMSC or hFSSC secretome for 6 h. ***p < 0.001, when compared to SFM

### hFSSC secretome accelerated wound healing rate in rats

The Sr-90 radiation rat skin injury was treated with hFSSC secretome (Fig. 4a). As shown in Fig. 4b, we observed that skin damage occurred on 1–2 weeks and reached to the most serious radioactive injury on the second week. In addition, the lightest degree of erythema, desquamation, crusting, and minimal scar formation was observed in hFSSC secretome group. As shown in Fig. 4c, the fastest wound healing rate occurred in the hFSSC secretome group compared with the other two control groups. Moreover, on the seventh week after radiation, the most rapid wound healing rate was 96.3% in hFSSC secretome group, but hUCMSC secretome group reached to 71.4% and SFM group reached to 51.3%, respectively. The animal experiment results suggest that hFSSC secretome has the greatest potential to accelerate the radiation skin injury in rats.

**Fig. 4:** Effects of hFSSC secretome on wound healing induced by Sr-90 radiation. **a** Animal experiment design. **b** Gross morphological changes during wound occurring and healing. **c** The wound healing rate changes in rats after radiation. Note that the smallest wound area and the fastest wound healing rate occurred in the hFSSC secretome compared to the other two groups. hUCMSC, human umbilical cord mesenchymal stem cells; hFSSC, human fetal skin stem cell. *n* = 10/group; *p < 0.05, **p < 0.01when compared to PBS; ^##^*p* < 0.01 compared to hUCMSC secretome group; bar = 5 mm; data, mean ± SD

### hFSSC secretome promoted wound healing quality and angiogenesis in rats

H&E staining results showed that hFSSC secretome group led to the largest number of cutaneous appendages, including hair follicles, sweat gland, and sebaceous glands (PBS, 4.7 ± 2.8; hUCMSC secretome, 22.3 ± 4.4; and hFSSC secretome, 43.1 ± 5.6/field 40×; Fig. 5a–d). IHC results showed that hFSSC secretome group had the greatest vessel number (i.e., α-SMA positive area) compared to the other two control groups (PBS, 3.6 ± 2.6; hUCMSC secretome, 11.5 ± 3.8; and hFSSC secretome, 24.6 ± 4.8/field 40×; Fig. 5e–h). The histological results suggest that hFSSC secretome significantly promoted the wound healing quality and angiogenesis of radiation skin injury.

**Fig. 5:** Effects of hFSSC secretome on wound healing quality and angiogenesis. **a**–**c** H&E staining evaluation on cross sections of healed tissue. **d** Number of cutaneous appendages (hair follicles, sweat gland, and sebaceous glands)/field (40×) in the healed tissue. **e**–**g** α-SMA-positive cells/field (100×) in the healing tissue. **h** Number of vessels/field (100×) in the healing tissue. Note that *n* = 10/group; *p < 0.05, **p < 0.001; bar = 1 mm; data, mean ± SD

### hFSSC secretome regulated gene and protein expression in wound healing tissue

Gene study results showed that hFSSC secretome group had the lowest relative expression levels of Col1A2 and TGF-β1, but with the highest expression levels of Col3A1 and TGF-β3 compared to the other two control groups, in consistent with proteins expression (Fig. 6a, c). The expression level of angiogenesis-related genes, including Ang-1, Ang-2, VEGF, and PLGF, was significantly increased in hFSSC secretome group when compared to the other control group, as consistent with protein expression (Fig. 6b, c). These results suggest that hFSSC secretome promotes the radioactive wound healing through activating the expression of specific genes which are related with the fetal skin regeneration and angiogenesis.

**Fig. 6:** Effects of hFSSC secretome on wound healing quality and angiogenesis-related gene and protein expression. **a** Col1A2, Col3A1, TGF-β1, and TGF-β3 gene expression. **b** Ang-1, Ang-2, VEGF, and PLGF gene expression. **c** Col1A2, Col3A1, TGF-β1, TGF-β3, Ang-1, Ang-2, VEGF, and PLGF protein expression. TGF-β1, transforming growth factor-beta 1; TGF-β3, transforming growth factor-beta 3; VEGF, vascular endothelial growth factor; PLGF, placental growth factor. *p < 0.05, **p < 0.01, ***p < 0.001; mean ± SD

## Discussion

To the best of our knowledge, this is the first time of the administration of hFSSC secretome to treat the radiation skin injury in rats. We found that hFSSC secretome accelerated wound closure rate and enhanced wound healing quality, and significantly promoted angiogenesis both in vivo and in vitro. Moreover, hFSSC secretome provided an even stronger cell therapeutic potential in comparison to hUCMSC secretome.

Stem cells and their secretome play an important role in skin repair and regeneration [20, 21]. Generally, stem cells secrete various growth factors [22], pro-inflammatory and anti-inflammatory cytokines [23], and other cytokines which could enhance the wound healing effect. Moreover, the healed tissue in stem cell groups showed the faster wound closure [24], less granulation tissue area [25], and more neovascularization than that in control group [26]. These studies demonstrated that stem cells exert beneficial effects on the damaged tissue due to their ability of secreting the soluble factors, rather than their capacity to differentiate into the needed cells [27, 28]. Finding suitable cell sources is one of the main challenges in regenerative medicine [29–31]. In the present study, we selected the stem cells derived from human fetal tissue, which have greater clinical therapeutic potential. CD73, CD90, and CD105 are common cell surface markers of mesenchymal stem cells [32], while Oct4 and Sox2 are the classical markers of embryonic stem cells [33]. In this study, positive expressions of CD73, CD90, CD105, Oct4, and Sox2 were observed in hFSSC which indicated that hFSSC presented with the characteristics of both MSC and embryonic stem cell (ESC).

Stem cell may secrete many factors to promote angiogenesis efficiently [34, 35], such as TGF-β1, VEGF, hepatocyte growth factor (HGF), platelet-derived growth factors (PDGF), and insulin-like growth factors (IGF), which can trigger angiogenesis [36, 37]. It has been reported that Wharton’s jelly-derived MSCs could promote neovascularization and function as perivascular precursor cells [38]. In other investigations, adipose-derived MSCs secrete angiogenic cytokines which increased neovascularization and enhanced wound healing in rat injured tissues [35]. To validate our results, we used an HUVEC model to study the effects of hFSSC secretome on cell proliferation and tube formation, and Sr-90 radiation-induced skin injury rat model to test the angiogenesis-related gene expression in healed tissues. Ki-67 was reported to be a common cellular proliferation marker [39]. Our study showed the highest level of Ki-67 in hFSSC secretome group (Fig. 2a, b). In addition, the proliferation curves of HUVEC also indicated that hFSSC secretome could promote HUVEC proliferation significantly. To determine the angiogenesis effects of hFSSC secretome, we first examined the tube formation in different groups. The results showed the most tube formation in hFSSC secretome group. In addition, the expression of angiogenesis-related genes, including Ang-1, Ang-2, VEGF, and PLGF, was significantly increased in vivo (Fig. 6). Although hUCMSCs have been reported to be effective in promoting angiogenesis [40, 41], hFSSC secretome was found superior to hUCMSC secretome in our experiments. We observed that hFSSC secretome has enormous capacity in angiogenesis which is beneficial to accelerate wound closure rate and enhance wound healing quality (Figs. 4 and 5).

hFSSCs can promote fetal-like skin regeneration in rats with radiation-induced skin injury. A study has shown that the fetal skin contains a higher ratio of collagen type III to collagen type I than adult skin [42], as well as a different profile of proteoglycan and glycosaminoglycan synthesis [43]. It is probable that both the fetal skin cells and the ECM they synthesize are critical in scarless repair [44]. In this study, the expression of Col3A1 was significantly increased and the expression of Col1A2 was statistically suppressed in hFSSC secretome group than that in the other two groups (Fig. 6a, c). As a result, the ratio of Col3A1/Col1A2 was increased in the hFSSC secretome treatment group which could match with that of fetal skin characteristics. On the other hand, TGF-β1, TGF-β2, and TGF-β3 ligands have been implicated in the ontogenetic transition from scarless fetal repair to adult repair with scar [45]. Specifically, TGF-β1 and TGF-β2 may promote scar formation, whereas TGF-β3 may reduce scarring [43]. The addition of exogenous TGF-β1 to normally scarless fetal wounds results in scar, while neutralizing antibodies against TGF-β1 and TGF-β2 in adult wounds decreases scarring [46]. In this study, we found that the ratio of TGF-β3/TGF-β1 was increased which is similar to fetal skin. These results above demonstrated that hFSSC secretome can induce scarless wound repair by activating fetal-like skin regeneration.

## Conclusions

In conclusion, hFSSC has great wound healing capabilities to treat the radiation skin injury in rats. Our data indicated that hFSSC promoted wound healing quality and angiogenesis. Moreover, we found that the healed tissue of hFSSC secretome closely resembled the fetal skin. hFSSC secretome may serve as the basis of cell-free therapeutic approach for optimal wound healing.

## Supplementary information

**Additional file 1: Figure S1. a** Migration of HUVECs into the scratch wound after 0, 24 h of culture with SFM, hUCMSC secretome, and hFSSC secretome in the scratch wound assay. **b** Migration distance of HUVECs movement after 24 h. The migration distance of movement was significantly greater for HUVECs cultured with hFSSC secretome compared with the other two control groups. Bar = 200 μm, ** *p* < 0.01. **Figure S2.** Fractionation of the ASC-CM components using AKTA protein chromatography. **a** SFM, four peaks identified. **b** hUCMSC secretome, four peaks identified. **c** hFSSC secretome, five peaks identified. Note that hUCMSC secretome group had one more peaks appeared at retention volumes of 40 ml than the other two control groups. **Figure S3.** The dose response study on hFSSC secretome treatment in rats after radiation. Note that the administered secretome dose (1 mg secretome per 1 ml injection) was suitable in hFSSC secretome groups.*p < 0.05, **p < 0.01. (DOCX 3968 kb)

**Additional file 2: Table S1.** Primers used for real time PCR. (DOCX 23 kb)

## Data Availability

The datasets used and/or analyzed during the present study are available from the corresponding author on reasonable request.

## Abbreviations

Ang-1: Angiotensin 1
Ang-2: Angiotensin 2
BSA: Bovine serum albumin
Col1A2: Collagen type I α 2
Col3A1: Collagen type III α 1
ECM: Extracellular matrix
ESC: Embryonic stem cell
hFSSC: Human fetal skin-derived stem cell
HGF: Hepatocyte growth factor
HLA-G: Human leukocyte antigen G
hUCMSC: Human umbilical cord mesenchymal stem cell
HUVEC: Human umbilical vein endothelial cell
IF: Immunofluorescence staining
IGF: Insulin-like growth factors
IHC: Immunohistochemistry
MSC: Mesenchymal stem cell
PDGF: Platelet-derived growth factors
PLGF: Placental growth factor
SFM: Serum-free medium
TGF-β: Transforming growth factor β
TGF-β1: Transforming growth factor β1
TGF-β3: Transforming growth factor β3
VEGF: Vascular endothelial growth factor
α-SMA: Alpha-smooth muscle actin
